The article "Network Toxicology Guided Mechanism Study on the Association between Thyroid Function and Exposures to Polychlorinated Biphenyls Mixture" was published in 2022. Journal: Biomed Res Int.

# Network Toxicology Guided Mechanism Study on the Association between Thyroid Function and Exposures to Polychlorinated Biphenyls Mixture

**DOI:** 10.1155/2022/2394398

**Published:** 2022-09-27

**Authors:** Chunxia Li, Hong Xing, Qiaoyu He, Jing Liu, Hong Liu, Yue Li, Xiaopeng Chen

**Affiliations:** State Key Laboratory of Component-Based Chinese Medicine, Tianjin University of Traditional Chinese, Tianjin 301617, China

## Abstract

Polychlorinated biphenyls (PCBs) are persistent and highly toxic pollutants, which can accumulate in organisms and produce toxic effects, especially damaging the function of thyroid hormones. So far, the molecular mechanism of PCBs mixture and their metabolites interfering with thyroid hormones has not been studied thoroughly except for individual compounds. In this study, PubMed, Web of Science, and STITCH databases were used to search PCBs and their corresponding target proteins. The intersection of PCBs and thyroid hormone dysfunction target proteins was obtained from GeneCards. The “compounds-targets-pathways” network was constructed by Cytoscape software. And KEGG and Go analyses were performed for key targets. Finally, molecular docking was used to verify the binding effect. Four major active components, five key targets, and 10 kernel pathways were successfully screened by constructing the network. Functional enrichment analysis showed that the interference was mediated by cancer, proteoglycans, PI3K-Akt, thyroid hormone, and FoxO signaling pathways. The molecular docking results showed that the binding energies were less than -5 kcal·mol^−1^. PCBs and their metabolites may act on the key targets of MAPK3, MAPK1, RXRA, PIK3R1, and TP53. The toxic effect of sulfated and methyl sulfone PCBs is greater. The method of screening targets based on the simultaneous action of multiple PCBs can provide a reference for other research. The targets were not found in previous metabolite toxicity studies. It also provides a bridge for the toxic effects and experimental research of PCBs and their metabolites in the future.

## 1. Introduction

With the rapid development of the electronic products market in the world, the growth of electronic waste has become a global environmental health issue [1]. The removal of these wastes will inevitably release polychlorinated biphenyls (PCBs) and other toxic substances into the environment. In the 1970s, PCBs were a class of industrial compounds, which were widely used in products such as electrical insulators, coatings, and adhesives [2]. They consist of two linked benzene rings with varying degrees of chlorination, producing 209 different congeners. PCBs are listed under the Stockholm Convention on Persistent Organic Pollutants [3].

The article "Network Toxicology Guided Mechanism Study on the Association between Thyroid Function and Exposures to Polychlorinated Biphenyls Mixture" was published in 2022. Journal: Biomed Res Int.

Although they have been banned, they exist in soil, sediment, and biota as persistent organic pollutants (POP) [4]. PCB exposure has been reported to be associated with thyroid dysfunction (hypothyroidism) in mammals. Studies have shown that exposure to PCBs and their metabolites in the environment can interfere with the function of thyroid hormones (THs) and disrupt gene transcription mediated by thyroid receptors, resulting in thyroid hormone dysfunction that can seriously affect the basal metabolism, normal growth, and development of the organism [5]. It is worth noting that it not only regulates the physiological process of normal cells but also stimulates the proliferation of cancer cells through the imbalance of molecular and signal pathways. PCBs are structurally similar to thyroid hormone, and their binding characteristics are similar to thyroid hormone. The main thyroid hormones produced by the thyroid gland are thyroxine (T4), 3, 5, 30-triiodothyronine (T3), and reverse 3, 5, 30-triiodothyronine (rT3), which are controlled by thyroid-stimulating hormone (TSH) [6]. Some studies have shown that the mechanism of polychlorinated biphenyls induced hypothyroidism may be the replacement of thyroid hormone combined with the transporter in the blood, which increase the effect of coupling reaction and enhance the elimination of thyroid hormone (TH) [7]. PCB poisoning then inhibits the activity of choline acetyltransferase (ChAT) in the hippocampus and basal forebrain of rats [8]. PCBs can bind to cytosolic aromatic hydrocarbon (AH) receptor, thyroid hormone receptor, and serum thyroid hormone-binding transthyroxine protein, which leads to thyroid dysfunction, and interferes with thyroid hormone (TH) level and its signal transduction, affects brain development, and even produces neurotoxicity [9–11].

It is important to note that the metabolites of PCBs in humans, including hydroxylated, sulfated, and methyl sulfone PCBs, are more toxic than their parent PCBs. These metabolites have harmful effects on reproductive processes, the endocrine system, and brain function in humans [12]. Electrophoretic mobility shift assay (EMSA) was performed to examine thyroid hormone receptor-thyroid hormone response element (TR-TRE) bindings under exposure of 4'-OH-2',3,3',4',5'-pentachloro biphenyl (4'-OH-PCB-106). In EMSA, the thyroid hormone receptor (TR) is separated from the malic enzyme (ME)-TRE by 4'-OH-PCB-106. The findings suggest that hydroxylated PCBs (OH-PCB) may disrupt TR mediated transcription on natural promoters [13]. In some studies, the luciferase reporter gene was used to determine that lower chlorinated polychlorinated biphenyls (LC-PCB) sulfates have a higher binding effect than its corresponding OH-PCB precursor. It was found that LC-PCB sulfates have a better binding effect on thyroid hormone receptor alpha (THRA). The signaling pathway showed agonistic activity, and the mechanism may be the destruction effect of the thyroid hormone (TH) system induced by LC-PCB sulfates [14].

The article "Network Toxicology Guided Mechanism Study on the Association between Thyroid Function and Exposures to Polychlorinated Biphenyls Mixture" was published in 2022. Journal: Biomed Res Int.

PCBs prototypes and their metabolites exist in the form of mixtures in the environment. At present, the research on PCB toxicity mainly starts from monomers, but in reality, PCB exists in the form of a mixture, so it is necessary to use a holistic idea and method to explore the mechanism of PCBs homologs and metabolites interfering with thyroid hormone disorder, to evaluate the potential health risk.

Network toxicology is a new discipline based on network theory and the principles of systems biology. It is considered to be an effective tool for systematically revealing complex network relationships. It can reveal the complex overall biological network relationships between “toxicity-targets-components-drug” and provide a new perspective for analyzing and predicting the functional mechanisms of components [15]. PCBs homolog has 209 components, which have the characteristics of multicomponent, multitarget, and multichannel synergy. It is an exploration that we use network toxicology on PCBs homologs. Finding the key targets and pathways of PCBs interfering with thyroid hormone endocrine disorder can reveal the action mechanism based on multiple components and targets. Applying network toxicology to environmental toxicology also provides a basis for further study on the toxicological mechanism of thyroid endocrine disorder caused by small molecular organic pollutants.

Molecular docking is an important approach in structural molecular biology and computer-aided design of new drugs, which can further predict the recognition and interaction patterns between components and their predicted targets [16–19].

To fully understand the toxicity of phototype and metabolites (prototype, hydroxylated, sulfated, and methyl sulfonated) of PCBs on human thyroid dysfunction, the study explores their mechanism of action based on network pharmacology and molecular docking systematically, which was shown in Figure 1. We found the typical toxic PCBs interfering with thyroid hormone through literature research; predicted, analyzed, and screened their key targets; uncovered the signal pathways by using relevant databases and software; studied the molecular mechanism of PCBs interfering with thyroid hormone from an overall perspective; and verified the molecular role between PCBs prototype and metabolites and target receptors through molecular docking.

The article "Network Toxicology Guided Mechanism Study on the Association between Thyroid Function and Exposures to Polychlorinated Biphenyls Mixture" was published in 2022. Journal: Biomed Res Int.

## 2. Materials and Methods

### 2.1. Software and Database

The databases used are as follows: PubMed, Web of Science and PharmMapper database (http://www.lilab-ecust.cn/pharmmapper/),UniProtdatabase (https://www.uniprot.org/), PubChem (https://pubchem.ncbi.nlm.nih.gov/), STRING database (https://string-db.org/), David database 6.8 (https://david.ncifcrf.gov/), STITCH database (http://stitch.embl.de/), Swiss Target Prediction (http://www.swisstargetprediction.ch/), SEA database (http://sea.edbc.org/), GeneCards database (https://www.GeneCards.org/), PDB database (https://www.rcsb.Org/), KEGG (https://www.kegg.jp/), and Venny 2.1 (http://bioinfogp.cnb.csic.es/tools/venny/index.html) online tool. The softwares used are as follows: Cytoscape 3.6.1, MGLTools-1.5.6, PyMOL software (http://pymol.org/2/), PLIP database: (https://projects.biotec.tu-dresden.de/plip-web/plip/index), and AutoDock Vina software (http://vina.scripps.edu/).

### 2.2. Screening of Active PCBs

To collect the active PCBs, PubMed and Web of Science databases were used to screen relevant research articles, the reference time is from 1987 to 2021, and the keywords “PCBs,” “thyroid hormone disorder,” “thyroid hormone,” and “thyroid” were used to look up the active components of PCBs related to thyroid hormone dysfunction manually (date: 2021.01.13-03.15).

### 2.3. Target Prediction of PCBs

Fourteen compounds in 2.2 were saved as 3D structures in SDF format and uploaded to the PharmMapper database. In the select targets set option, select “Homo sapiens” for target prediction, and use the UniProt database to correct disease targets and PCBs targets. Input the smiles structural formula of the compounds into STITCH, respectively, Swiss target prediction, and SEA databases. In the database, the species “Homo sapiens” was selected to retrieve, and the target was obtained and saved in the corresponding format. Finally, the target was summarized, and the duplicate items were deleted (date: 2021.03.15-03.24).

### 2.4. Target Prediction of Thyroid Disorder

GeneCards and PubMed databases were used to input “thyroid dysfunction” as the keyword, and the species “Homo sapiens” were selected for retrieval. Then, intersect and delete duplicate targets to obtain disease targets. UniProt database was used to correct disease targets (date: 2021.03.25-3.29).

### 2.5. Screening of Common Targets of PCBs and Disease

Venny 2.1 online tool was used to obtain the common targets of PCBs and diseases by entering the above Section 2.3 targets related to PCBs and thyroid dysfunction diseases. date: 2021.03.30-4.04).

### 2.6. Protein Interaction Network Construction and Kernel Target Screening

The intersection targets of “PCBs thyroid dysfunction” obtained in Section 2.5 were imported into the string database. In the model, select the species “Homo sapiens,” set the minimum interaction threshold to 0.400, hide the free nodes, and keep the default settings for other parameters. Then, import this network into Cytoscape 3.6.1 to build a protein-protein interaction (PPI) network and export excel. The kernel targets were selected according to the degree value ranking (date: 2021.04.06-04.15).

The article "Network Toxicology Guided Mechanism Study on the Association between Thyroid Function and Exposures to Polychlorinated Biphenyls Mixture" was published in 2022. Journal: Biomed Res Int.

### 2.7. Go Enrichment Analysis and KEGG Pathway Analysis

The key targets screened in Section 2.6 were imported into David 6.8 database, and the “Homo sapiens” species were selected. Go function enrichment analysis and KEGG pathway analysis were carried out on the predicted target genes. Click to select three entries of Go and KEGG entries, respectively, set the conditions of Benjamin <0.01 and count >5 for screening, and select the top 10 for mapping display, to further clarify the mechanism of polychlorinated biphenyls interfering with thyroid dysfunction (date: 2021.04.17-04.25).

### 2.8. Construction of “Components-Targets-Pathways” Network

To explore the main active components of PCBs, the selected active components, targets, and signaling pathways of PCBs were used to construct the “components-targets-pathways” network visualization by using the software Cytoscape 3.6.1 (date: 2021.04.26-04.29).

### 2.9. Docking Verification of PCBs and their Metabolites with Kernel Target Genes

When the conformation of ligand and receptor is stable, the lower the energy, the greater the binding effect. Select PCBs (PCB-118, PCB-126, PCB-180, PCB-146 and corresponding hydroxylated, sulfated, and methyl sulfone metabolites) with the highest degree value in the “components-targets-pathways” network and the target genes (MAPK3, MAPK1, RXRA, PIK3R1, and TP53) with the highest degree value in the PPI network for molecular docking. The 3D structures of the PCBs were obtained by Chem3D 19.0 software and optimized by the MM2 function to obtain the best structure. Protein crystals holding core targets were downloaded using the RCSB PDB database (http://www.rcsb.org/) [20]. Water and self-ligands were removed by the PyMOL software. Protein crystals import structures into AutoDock for processes such as hydrogenation, calculation of total charge, and addition of atom types. AutoDock Vina was used for molecular docking [21], and each grid size is adjusted based on the minimum value of 40 for the number of points in *x*-dimension, *y*-dimension, and *z*-dimension. By adjusting the size of the box, the network wraps the whole protein for the next docking. PLIP database was used to check the interaction force, and PyMOL software was used for molecular docking visualization [22] (date: 2021.05.02-05.28).

The article "Network Toxicology Guided Mechanism Study on the Association between Thyroid Function and Exposures to Polychlorinated Biphenyls Mixture" was published in 2022. Journal: Biomed Res Int.

## 3. Results

### 3.1. Network Toxicology

#### 3.1.1. Screening of PCBs Related to Thyroid Dysfunction

Experimental evidence shows that exposure to halogenated compounds such as PCBs may interfere with the endocrine system, especially thyroid function [23, 24]. According to the laboratory parameters, the geometric mean of serum concentrations of PCB-118, 138, 153, and 180 in patients with thyroid disease was higher than those in patients without thyroid disease [25]. Continuous exposure to low doses of PCB-118 can seriously damage thyroid structure, significantly reduce the concentration of serum thyroid hormone, and inhibit the expression of key genes such as sodium/iodide symporter (NIS) and thyroglobulin (TG) [26]. PCB-180 exposure affects the thyroid system by decreasing circulating thyroid hormone levels, altering thyroid weight and histology, as well as increasing liver expression (mRNA and protein) and activity of UDP-glucuronyltransferases (UGTs), responsible for thyroid hormone elimination, among others [27]. The hydroxyl metabolite of PCB-180 replaces the thyroid hormone in transthyretin (TTR), which further leads to hypothyroidism [28]. It has been reported that in a nested case-control study conducted in Norway, high concentrations of PCB-146, 153, and moderately chlorinated PCBs were associated with thyroid cancer [29]. Other studies have shown that significant interaction and positive correlation with thyroid cancer were observed in the homologs of PCB-138, 158, 146, 153, and 183 [30]. The mechanism of PCB-153 interfering with thyroid hormone homeostasis may reduce THS through thyroid hormone receptors [31]. PCB-105, 118, and 126 have tissue-specific and gene-specific effects on thyroid hormone signaling during development [32]. Based on the toxicological experiments, PCB 95 exposure caused a dose-dependent (*p* < 0.001) decrease in serum thyroxine (T4) levels. Morphological analysis of the thyroid showed that the colloidal area of rats treated with PCB-95 decreased and the proliferation of thyroid epithelial cells increased. The results suggest that the hypothalamus-pituitary-thyroid (HPT) axis appears to be a target of ortho-substituted PCBs [33]. PCB-126 significantly increased the mRNA expression of TPO and TG genes, indicating that PCB-126 can directly affect the synthesis and secretion of thyroid hormone, which may disturb the endocrine function of laying hens' thyroid [34]. The pharmacokinetic study suggests that the primary mode of action of PCB-126 on the HPT axis in the adult male Sprague Dawley rat is increased phase II metabolism of thyroxine, presumably mediated by arylhydrocarbon receptor (AhR), and the dose-response characteristics of PCB-126 induced perturbations in the HP Taxis are complex and nonlinear [35]. Bivariate analysis adjusted for total serum lipids showed a statistically significant positive correlation between free thyroxine and highly correlated PCB-153, 170, 171, 156, and 180 [36]. PCB-99 can increase the glycolaldehyde fixation and bile excretion of thyroxine, which is different from those compounds that promote the disappearance of thyroxine in serum [37]. It has been studied that early-weaned male rats were given early PCB-95. Compared with the control group, the concentrations of serum thyroxine, triiodothyronine, and thyroxine in the PCB-95 group decreased. Results imply that PCB-95 may act as a disruptor of the developmental hypothalamic–pituitary–thyroid axis hypothyroidism is caused by PCB-95 [38]. Based on the homologs of PCBs reported in the literature, we selected PCB-95, PCB-99, PCB-105, PCB-118, PCB-126, PCB-138, PCB-146, PCB-153, PCB-156, PCB-158, PCB-170, PCB-171, PCB-180, and PCB-183 as the research objects. With the help of PubChem, the 3D structures of the above 14 PCBs homologs were queried and saved, respectively, in SDF format. The name and SMILE structural formula of 14 compounds are inquired using the database PubChem, as shown in Table 1.

The article "Network Toxicology Guided Mechanism Study on the Association between Thyroid Function and Exposures to Polychlorinated Biphenyls Mixture" was published in 2022. Journal: Biomed Res Int.

#### 3.1.2. Screening of PCBs Related Targets

The smile structural formulas of the 14 PCBs were input into the Swiss target prediction database, SEA database, and STITCH database, respectively. With “Homo sapiens” as the screening condition, 1, 22, and 29 predicted targets were obtained. Then, input the 3D structures of the above compounds into the PharmMapper database one by one, select “Homo sapiens” in the select targets set option, and summarize 183 related targets of all compounds. Two hundred and nineteen predicted target genes were obtained by combining the above targets and deleting repeats.

#### 3.1.3. Screening of Targets Related to Thyroid Dysfunction

7,505 disease targets were screened by using “thyroid hormone dysfunction” as the keyword in the GeneCards database. The targets with a score value greater than the double median were selected as targets related to thyroid hormone dysfunction. The maximum score value of thyroid hormone dysfunction targets was 135.17, the minimum score value was 0.41, and the double median was 5.52. Therefore, 1,849 targets with scores bigger than 5.52 were selected as targets of thyroid hormone dysfunction. On the other hand, 1,306 targets of thyroid hormone dysfunction were obtained by using the PubMed database. 2,438 targets of thyroid hormone dysfunction were predicted by deleting duplicate items in total.

The article "Network Toxicology Guided Mechanism Study on the Association between Thyroid Function and Exposures to Polychlorinated Biphenyls Mixture" was published in 2022. Journal: Biomed Res Int.

#### 3.1.4. Target Intersection PPI Analysis

One hundred and forty intersection genes (Figure 2) were analyzed by string website and visualized by Cytoscape 3.6.1 software. The PPI network of PCBs interfering with thyroid function was obtained, and the core targets were screened. The degree value reflects the importance of the node in the network. According to the analysis results, 121 main nodes and 446 edges are obtained. In the PPI network, MAPK3, MAPK1, RXRA, PIK3R1, TP53, HSP90AA1, SRC, MAPK8, and MAPK14 are the top 9 nodes ranked according to the median value of 4 times 20 (Figure 3), that is, important targets for PCB disturbing thyroid function, which may play an important role in the process of PCB disturbing thyroid function.

#### 3.1.5. GO Function Enrichment Analysis

Using David 6.8 database to perform GO function enrichment analysis on 140 predicted target genes. Three GO items were selected, and a functional annotation chart was selected. A total of 614 items were selected. The dataset was established. One hundred and sixty-eight items were selected according to the conditions of *p* value <0.05, FDR<0.05, and Benjamin<0.01. The items of biological process, cell composition, and molecular function are 101, 51, and 16, respectively. The top 10 of each are selected for visualization. As shown in Figure 4, the target genes are significantly enriched in steroid hormone receptor activity, RNA polymerase II transcription factor activity, ligand-activated sequence-specific DNA binding, enzyme binding, protein tyrosine kinase activity, protein binding, and other molecular functions, steroid kinases-mediated signaling pathway, RNA polymerase II promoter transcription initiation, and negative regulation of apoptosis process. Studies have found that targets and biological functions form a complex biological network; one target can regulate a variety of biological functions; and a biological function also has multiple target enrichment [39]. It suggests that PCBs interfere with thyroid dysfunction by regulating multiple targets and a variety of biological functions.

#### 3.1.6. KEGG Pathway Analysis

David 6.8 database was used to analyze the KEGG pathway of 140 predicted target genes. According to *p* value <0.05, FDR<0.05, and Benjamin <0.01, a total of 77 pathways were screened out. The top 10 related signaling pathways are shown in Table 2, including tumor, proteoglycan in cancer, prostate cancer, PI3K-Akt signaling pathway, Ras signaling pathway, thyroid hormone signaling pathway, prolactin signaling pathway, progesterone-mediated oocyte maturation, pancreatic cancer, and FoxO signaling pathways. The pathways often have multiple target relationships with complex networks, indicating that PCBs may regulate the pathways based on the 140 targets to interfere with thyroid hormone dysfunction. The thyroid signal pathway is gained through the KEGG database to obtain the target distribution of PCB in the thyroid hormone signaling pathway. As shown in Figure 5, the red border is the potential target genes, and the arrow indicates the upstream and downstream relationship between genes.

The article "Network Toxicology Guided Mechanism Study on the Association between Thyroid Function and Exposures to Polychlorinated Biphenyls Mixture" was published in 2022. Journal: Biomed Res Int.

#### 3.1.7. “Components-Targets-Pathways” Network Analysis

The selected 14 PCBs, 115 targets, 10 signaling pathways, and diseases are visualized by using Cytoscape 3.6.1 software to construct a “components-targets-pathways” network, as shown in Figure 6. It is interesting to find that there is little difference in the degree values of PCBs homologs, presumably because of their similar structures. PCB-118 (degree =126), PCB-126 (degree =124), PCB-180 (degree =123), and PCB-146 (degree =121) have high connectivity in the network, suggesting that these compounds may be the main active components of PCBs interfering with thyroid hormone dysfunction. Based on the results, we selected the four active components in the following molecular docking.

### 3.2. Molecular Docking

Molecular docking is to place small-molecule ligands in the binding region of macromolecular receptors by computer simulation and then calculate the physical and chemical parameters to predict the binding affinity between them. The docking energy is determined by the ligand-receptor affinity score function. In this study, the target proteins with the highest screening degree of the PPI network were used for molecular docking verification with the active PCBs with the highest screening degree of the “components-targets-pathways” network. Meanwhile, the hydroxylated, sulfated, and methyl sulfone metabolites of the main active PCBs were selected for molecular docking with the kernel target proteins. PCB-126 had no reference metabolite data. Metabolite conversion is shown in Figure 7.

Based on the degree ranking, the top four active components from the “components-targets -pathways” network and the top five core targets from the PPI network were verified by molecular docking. The RCSB PDB database, powered by the protein database, contains archived information about the three-dimensional shape of proteins, nucleic acids, and complex assemblies, helping researchers understand all aspects of biomedicine, from protein synthesis to health and disease. AutoDock Vina is an open-source molecular docking program, which can produce improved scoring functions. Therefore, we searched the PDB database for the top five potential targets, which were MAPK3 (PDB ID:6GES) [40], MAPK1(PDB ID:6SLG) [41], RXRA (PDB ID:6JNO) [42], PIK3R1(PDB ID:7JIS) [43], and TP53(PDB ID:5G4N) [44] and the top four compounds PCB-118, PCB-126, PCB-180, and PCB-146 with their three-dimensional structure and degree values. Using AutoDock Vina, we generated different sizes of mesh boxes, almost covering the entire favorable protein binding sites. Then, Discover Studio and PyMOL software were used to analyze the docking results. High-quality 3D and 2D structure maps of small molecules and proteins were made, while the corresponding protein residues and binding bonds were displayed. In addition, the binding data of the protein with its ligand were used as the baseline data of the control.

The article "Network Toxicology Guided Mechanism Study on the Association between Thyroid Function and Exposures to Polychlorinated Biphenyls Mixture" was published in 2022. Journal: Biomed Res Int.

As shown in Figure 8, 65 pairs of docking results were obtained. It can be concluded from the data that all binding energies are less than -5 kcal·mol^−1^, indicating a strong affinity and toxic effect of interfering with a thyroid hormone disorder. By comparing the binding energy, it was found that except that the binding energy of TP53 and 3-MeSO2-PCB-118 was lower than that of TP53 and its ligand, the binding energy of other proteins (MAPK1, MAPK3, RARX, and PIK3R1) with PCBs and metabolites was higher than that of its ligand. From low to high, the top three binding energies are RXRA (PDB ID: 6GNO) and 3-sulfate-PCB-118, PIK3R1 (PDB ID: 7JIS), and 3-MeSO_2_-PCB-118, MAPK3 (PDB ID: 6GES) and 3'-sulfate-PCB-180, which suggested that sulfated and methyl sulfonated PCBs had a strong effect on thyroid hormone signaling. The detailed information on target compound interaction obtained by docking simulation is shown in Figures 9 and 10.

The results show that the low binding energy between PCBs and target proteins means good affinity, which results in strong interference. It has been found that the binding energies of the sulfated and methyl sulfone PCBs metabolites are relatively low, suggesting that they bind better to proteins and may have greater toxicity. This may be because of the hydrogen bonds. According to the cluster analysis (Figure 8), in the heat map, RXRA, PIK3R1, MAKP3, and MAKP1 are clustered into one group, and TP53 is in another group. It indicates that RXRA, PIK3R1, MAKP3, and MAKP 1 are closely bound with compounds suggesting that PCBs and their metabolites have a strong endocrine disrupting effect on thyroid hormones.

As shown in Figure 10(a), the 6GES amino acid residues GLU-194 and ARG-104 participated in the hydrogen bond and PRO-193 in the hydrophobic interaction between 3'-sulfate-PCB-180 and ligand. Among them, 3-MeSO2-PCB-118 can bind to amino acid residue ASP-111 in 6SLG through a hydrogen bond and also has hydrophobic interaction with IEU-156, ILE-31, and VAL-39 (Figure 10(b). Among 3-MeSO2-PCB-118 can bind to amino acid residue PHE-439 and GLY-443 in 7JIS through a hydrogen bond, a hydrophobic interaction with TRP-305, and also has *Π*-stacking with TRP-305 (Figure 10(c)). Among 3-MeSO2-PCB-118 can bind to amino acid residue PHE-113 and TYR-116 in 5G4N through a hydrophobic interaction (Figure 10(d)). Among 3-sulfate-PCB-118, can bind to amino acid residue PHE-609 in 6JNO through hydrophobic interaction and also has halogen bond with PRO-812 (Figure 10(c)).

The article "Network Toxicology Guided Mechanism Study on the Association between Thyroid Function and Exposures to Polychlorinated Biphenyls Mixture" was published in 2022. Journal: Biomed Res Int.

## 4. Discussion

There is evidence that PCBs have an important relationship with thyroid hormone disorders, which may be due to the similar structure of PCBs and thyroid-stimulating hormone (TSH), and high affinity with thyroid hormone-binding protein and metabolic enzymes [45]. After entering the organism, it can competitively bind thyroid transporters, thus interfering with the signaling pathway and producing thyroid hormone dysfunction [46]. There is experimental evidence that exposure to PCBs and other halogenated compounds may interfere with the endocrine system, especially thyroid function [47]. PCBs may also reduce the biological half-life of T4 by reducing the synthesis and secretion of T4 in the thyroid, and by activating glucuronyltransferase and the competitive binding carrier protein, thereby affecting the circulating thyroid hormones [48]. Data show that exposure to an e-waste dismantling environment may increase the toxicity of PCBs, and the release of pollutants from e-waste may lead to abnormal changes in thyroid hormone levels [49]. PCBs and halogen flame retardants (HFRs) are the main pollutants in the field of e-waste recovery, and exposure levels of PCBs and HFRs are harmful to the balance of human thyroid hormone [50]. Therefore, this experiment analyzed the molecular mechanism of PCBs and their metabolites destroying thyroid hormone disorder, including pharmacological targets, molecular functions, biological processes, and action pathways.

Five key targets were obtained through PPI network screening, namely, MAPK3, MAPK1, RXRA, PIK3R1, and TP53. Some studies have shown that these targets are related to thyroid diseases. As for important targets, protein mitogen-activated protein kinase 1 (MAPK1) is a protein kinase, which plays a crucial role in cell growth, differentiation, proliferation, survival, and inflammatory response [51]. Studies have shown that MAPK 1 is significantly upregulated in thyroid cancer cells cultured with high iodine, which promotes tumor growth [52]. Retinoid X receptor alpha (RXRA) is a member of the nuclear ligand-activated transcription factor family. It plays an important role in many cancers, such as human thyroid cancer, prostate cancer, and breast cancer. It can be achieved through Wnt/*β*-Catenin and RXRA enhancing human cholangiocarcinoma growth through simultaneous activation of Wnt/*β*-Catenin and nuclear factor-kappa B pathways (NF-kappa B) to promote cancer proliferation [53]. TP53 is a cancer suppressor protein, which plays an important role in the process of tumor regulation and human metabolism and development. Studies have shown that the abnormal increase of thyroid cancer is involved in the progress of tumors at the transcription and translation levels, suggesting that TP53 expression is involved in the occurrence and development of thyroid cancer [54].

The article "Network Toxicology Guided Mechanism Study on the Association between Thyroid Function and Exposures to Polychlorinated Biphenyls Mixture" was published in 2022. Journal: Biomed Res Int.

Through KEGG pathway analysis, we screened out kernel pathways such as a tumor, prostate cancer, PI3K-Akt signaling pathway, Ras signaling pathway, thyroid hormone signaling pathway, prolactin signaling pathway, pancreatic cancer, and FoxO signaling pathway, indicating that the underlying mechanisms of PCB interference in thyroid hormone dysfunction are mainly concentrated in the tumor, inflammation, and hormone levels. A PI3K-Akt signaling pathway is involved in cell proliferation, apoptosis, and cycle regulation. Studies have shown that hypothyroidism can inhibit the PI3K-Akt signaling pathway by inhibiting the expression of estrogen receptors and ultimately induce testicular cell apoptosis [55]. Thyroid cancer is the most common endocrine system cancer. Phosphatidylinositol 3-kinase-protein kinase B/Akt (PI3K-PKB/Akt) pathway is continuously activated by some abnormal receptor tyrosine kinase (RTK), and gene mutation occurs in its downstream effectors, leading to high cell proliferation including thyroid cancer [56]. Forkhead boxO (FoxO) is a subfamily of the forkhead transcription factor family, which plays an important role in determining cell fate. This subfamily is also considered to play a key role as a tumor suppressor in a variety of cancers [57]. The role of the thyroid hormone signal in the central nervous system is related to the development of thyroid disease symptoms. Thyroid hormone not only affects the target tissue through thyroid hormone receptor directly but also indirectly affects the target tissue by affecting the integration of sympathetic nerve signals in the target tissue [58]. Studies have shown that long-term exposure to environmental PCB can change the plasma thyroid hormone level, as well as gene expression related to thyroid hormone signal transduction, hypothalamus-pituitary-thyroid (HPT) axis, and liver metabolism leading to zebrafish dysplasia [59].

The article "Network Toxicology Guided Mechanism Study on the Association between Thyroid Function and Exposures to Polychlorinated Biphenyls Mixture" was published in 2022. Journal: Biomed Res Int.

To further clarify the research results of network toxicology, four prototype and nine metabolites of PCBs were calculated by molecular docking technology. The results showed that the docking binding energy was less than -5 kcal • mol^−1^, which verified the binding ability of targets screened by network toxicology. The results of molecular docking showed that the binding energy of sulfated and methyl sulfone metabolites of PCBs was relatively low compared with polychlorinated biphenyls and hydroxy polychlorinated biphenyls. The prototype cannot form hydrogen bonds, while some metabolites can indicate that the sulfated and methyl sulfone metabolites of PCBs bind well to protein and have greater toxicity. Studies have shown that PCB sulfate is a high-affinity ligand for human TTR, which is stronger than the binding ability of hydroxylated PCB metabolites to TTR [60, 61]. It also shows that it is consistent with the existing research, but the animal/human research specific to typical targets and metabolites needs to be further discussed.

Through data mining predicted by bioinformatics, we combine the exposure of organic chemical pollutants with molecular action pathways to better understand the toxic effects of exposure to organic pollutants on health. Use it to generate more innovative hypotheses, to design new experiments to establish the causal relationship between chemical environment and health, and to provide strategies for basic toxicity testing and verification [62]. The results still require further validation regarding the targeting of thyroid signaling by PCBs exposure. There are still some limitations to the current study. It is unclear how the overall results depend on the composition of the target organs/tissues/cells used in the database toxicology experiments [63]. In addition, the research method in the paper did not determine the quantitative aspects of the reaction between PCBs and specific targets (dose-response relationship), so future research will focus more on the quantitative aspects of the reaction between PCBs and specific targets [64]. Since data mining mainly depends on online sources (such as the TCMSP database) and the quality of existing interactions, without considering the individual sensitivity of exposed subjects, route of administration, duration, and individual drug metabolic rate, it should mainly be regarded as an insight into further in vivo and in vitro laboratory testing [65, 66]. The research methods also did not involve the differences in the toxicokinetics of different PCBs and did not investigate the addition/interaction effect of PCBs on specific targets.

The article "Network Toxicology Guided Mechanism Study on the Association between Thyroid Function and Exposures to Polychlorinated Biphenyls Mixture" was published in 2022. Journal: Biomed Res Int.

## 5. Conclusion

The relationship between the screened targets and PCB metabolites is first reported in the study, in which the targets were not found in the previous PCB metabolite toxicity studies. It means the network toxicology screening method, which is the target result of multiple PCB mixtures, is a useful tool and can provide new ideas for further research.

The study combined network toxicology with the molecular docking method. Through literature review, target prediction, network construction, functional enrichment analysis, and molecular docking analysis, the potential mechanism of PCBs interfering with thyroid hormones were predicted, clarified, and confirmed. In conclusion, PCBs can interfere with thyroid hormone dysfunction by regulating MAPK3, MAPK1, RXRA, PIK3R1, and other potential targets, as well as the cancer pathway, PI3K-Akt signaling pathway, thyroid hormone signaling pathway, prolactin signaling pathway, and FoxO signaling pathway. And the signal pathway shows that the screened core targets MAPK3, MAPK1, RXRA, PIK3R1, and TP53 are mainly enriched in the thyroid hormone pathway. The results of molecular docking show that the sulfated and methylsulfonated metabolites of PCBs have lower binding energy with target proteins, indicating that they are more toxic and thus have stronger endocrine disrupting effects on thyroid hormones. It is speculated that the structural formula contains oxygen, which makes it easier to form hydrogen bonds and a more stable binding force. This study preliminarily analyzed the molecular mechanism of PCBs and their metabolites interfering with thyroid hormone dysfunction, but further experimental verification is still needed. The findings provide a theoretical basis for further understanding the interference of PCBs and their metabolites on thyroid hormone dysfunction. Follow-up experiments will further study the impact of exposure to PCBs and their metabolites on thyroid hormone disorders.

## Figures and Tables

**Figure 1:** General workflow of network toxicology and molecular docking in the study.

**Figure 2:** Venn diagram of PCBs and thyroid hormone dysfunction targets. The diagram was built using Venny 2.1 online tool (http://bioinfogp.cnb.csic.es/tools/venny/) according to the data from the STRING database.

**Figure 3:** PPI network of PCBs interfering with thyroid hormone function. The PPI network was built using Cytoscape software 3.6.1 (http://cytoscape.org/) according to the data from the STRING database. The larger the node is, the more orange the color is, indicating that the target is more important in the network, the closer to the target in the inner circle, the more important the target is, the closer to the target in the inner circle, the more important the target is.

The article "Network Toxicology Guided Mechanism Study on the Association between Thyroid Function and Exposures to Polychlorinated Biphenyls Mixture" was published in 2022. Journal: Biomed Res Int.

**Figure 4:** Go (BP MF CC) function enrichment analysis diagram. The diagram was built using bioinformatics online tool (http://www.bioinformatics.com.cn/) according to the data from the DAVID 6.8 database. BP: biological process; MF: molecular function; CC: cellular component.

**Figure 5:** The target distribution of PCB in the thyroid hormone signaling pathway. The diagram was built using the KEGG database (https://www.kegg.jp/) (red rectangle indicating potential targets: GSK3B, MAP2K1, THRB, THRA, PDPK1, SRC, PIK3R1, ESR1, RXRA, and TP53.)

**Figure 6:** “Components-targets-pathways” network diagram. The network diagram was built using Cytoscape software 3.6.1. (https://cytoscape.org/). (The purple box represents PCBs pollutants, the blue box represents the chemical components of PCBs pollutants related to thyroid dyscalculia, the green box represents intersection targets, and the red box represents key pathways. Grey lines represent interactions).

**Figure 7:** Transformation pathway of three metabolites of PCBs in the human body (CYPs: cytochrome P450 enzymes; SULTs: sulfotransferases; MeSO_2_: methyl sulfone).

**Figure 8:** Heat map of the molecular docking energy scoring. The heat map was built using MeV software (http://mev.tm4.org/) (the closer the color is to blue, the better the binding ability.)

**Figure 9:** The 3D view of the molecular docking pattern of each protein with its ligand. The 3D pattern of target interaction was marked by PyMOL software (https://pymol.org/2/), PLIP database (https://projects.biotec.tu-dresden.de/plip-web/plip/index), and AutoDock Vina software (https://vina.scripps.edu/) (yellow dotted line: hydrogen bond; red dotted line: hydrophobic interaction; green dotted line: *Π*-stacking; purple dotted line: halogen bonds; blue dotted line: salt bridges. (a) 6GES, (b) 6SLG, (c) 7JIS, (d) 5G4N, (e) 6JNO; 3D: 3-dimensional).

**Figure 10:** The 3D visual analysis results of molecular docking of PCBs metabolite with key target proteins. The 3D visual analysis results of molecular docking were using PyMOL software (https://http://pymol.org/2/), PLIP database (https://projects.biotec.tu-dresden.de/plip-web/plip/index), and AutoDock Vina software (http://vina.scripps.edu/) (yellow dotted line: hydrogen bond; red dotted line: hydrophobic interaction; green dotted line: *Π*-stacking; purple dotted line: halogen bonds; blue dotted line: salt bridges. (a) 6GES and 3'-sulfate-PCB-180, (b) 6SLG and 3-MeSO2-PCB-118, (c) 7JIS and 3-MeSO2-PCB-118, (d) 5G4N and 3-MeSO2-PCB-118, (e) 6JNO and 3-sulfate-PCB-118; 3D: three-dimensional).

The article "Network Toxicology Guided Mechanism Study on the Association between Thyroid Function and Exposures to Polychlorinated Biphenyls Mixture" was published in 2022. Journal: Biomed Res Int.

**Table 1:** Homologous information of PCBs.

Compounds	Name	SMILES structure form
PCB-95	2,2',3,5',6-pentachlorobiphenyl	c_1_ = cc(=c(c = c_1_cl)c_2_ = c(c = cc(=c_2_cl)cl)cl)cl
PCB-99	2,2',4,4',5-pentachlorobiphenyl	c_1_ = cc(=c(c = c_1_cl)cl)c_2_ = cc(=c(c = c_2_cl)cl)cl
PCB-105	2,3,3',4,4'-pentachlorobiphenyl	c_1_ = cc(=c(c = c_1_c_2_ = c(c(=c(c = c_2_)cl)cl)cl)cl)cl
PCB-118	2,3',4,4',5-pentachlorobiphenyl	c_1_ = cc(=c(c = c_1_c_2_ = cc(=c(c = c_2_clcl)cl)cl)cl
PCB-126	3,3',4,4,5- pentachlorobiphenyl	c_1_ = cc(=c(c = c_1_c_2_ = cc(=c(c(=c_2_)cl)cl)cl)cl)cl
PCB-138	2,2',3,4,4',5'-hexachlorobiphenyl	c_1_ = cc(=c(c(=c_1_c_2_ = cc(=c(c = c_2_ cl)cl)cl)cl)cl)cl
PCB-146	2,2',3,4',5,5'-hexachlorobiphenyl	c_1_ = c(c = c(c(=c_1_c_2_ = cc(=c(c = c_2_ cl)cl)cl)cl)cl)cl
PCB-153	2,2',4,4',5,5'-hexachlorobiphenyl	c_1_ = c(c(=cc (=c_1_cl)cl)cl)c_2_ = cc(=c(c = c_2_ cl)cl)cl)cl
PCB-156	2,3,3',4,4',5-hexachlorobiphenyl	c_1_ = cc(=c(c = c_1_c_2_ = cc(=c(c(=c_2_ cl)cl)cl)cl)cl)cl
PCB-158	2,3,3',4,4',6-hexachlorobiphenyl	c_1_ = cc(=c(c = c_1_c_2_ = c(c(=c(c = c_2_ cl)cl)cl)cl)cl)cl
PCB-170	2,2',3,3',4,4',5-heptachlorobiphenyl	c_1_ = cc(=c(c(=c_1_c_2_ = cc(=c(c(=c_2_ cl)cl)cl)cl)cl)cl)cl
PCB-171	2,2',3,3',4,4',6-heptachlorobiphenyl	c_1_ = cc(=c(c(=c_1_c_2_ = c(c(=c(c = c_2_ cl)cl)cl)cl)cl)cl)cl
PCB-180	2,2',3,4,4',5,5'-heptachlorobiphenyl	c_1_ = c(c(=cc(=c_1_cl)cl)cl)c_2_ = cc(=c(c(=c_2_ cl)cl)cl)cl
PCB-183	2,2',3,4,4',5',6-heptachlorobiphenyl	c_1_ = c(c(=cc(=c_1_cl)cl)cl)c_2_ = c(c(=c(c = c_2_ cl)cl)cl)cl

**Table 2:** Top 10 pathways of KEGG.

KEGG	Description	*p* value	Target protein
hsa05200	Pathways in cancer	2.77E-20	GSK3B, GSTP1, XIAP, PIK3R1, EGFR, PIK3CG, IGF1R, RXRB, MAPK8, CASP8, RXRA, CASP3, AKT2, ABL1, MAPK1, PRKACA, MAPK3, TGFB2, MAP2K1, HSP90AA1, MMP2, IGF1, TGFBR1, PGF, MAPK10, AR, BMP2, RAD51, KIT, CDK2, RARA, MDM2, RARB, PPARG, MET, TP53, FGFR2, FGFR1, BCL2L1, PPARD
hsa05205	Proteoglycans in cancer	2.64E-15	SRC, PIK3R1, EGFR, PIK3CG, SLC9A1, IGF1R, ERBB4, CASP3, AKT2, KDR, MAPK1, PRKACA, MAPK3, TGFB2, MAP2K1, PDPK1, MMP2, PTPN11, IGF1, MAPK14, ESR1, PPP1CA, MDM2, MET, TP53, FGFR1
hsa05215	Prostate cancer	4.55E-15	GSK3B, MAP2K1, HSP90AA1, PDPK1, PIK3R1, IGF1, EGFR, PIK3CG, IGF1R, AR, CREB1, AKT2, CDK2, MDM2, MAPK1, TP53, FGFR2, FGFR1, MAPK3
hsa04151	PI3K-Akt signaling pathway	2.89E-12	GSK3B, PIK3R1, EGFR, PIK3CG, IGF1R, RXRA, AKT2, KDR, MAPK1, JAK2, MAPK3, MAP2K1, HSP90AA1, SYK, PDPK1, INSR, IGF1, IL2, PGF, CREB1, KIT, CDK2, MDM2, TEK, MET, TP53, FGFR2, FGFR1, BCL2L1
hsa04014	Ras signaling pathway	3.36E-12	MAP2K1, INSR, PLA2G2A, PTPN11, PIK3R1, IGF1, EGFR, PGF, PIK3CG, IGF1R, MAPK10, MAPK8, AKT2, KIT, KDR, ABL1, MAPK1, TEK, PRKACA, MET, FGFR2, FGFR1, BCL2L1, MAPK3
hsa04919	Thyroid hormone signaling pathway	7.42E-12	GSK3B, MAP2K1, THRB, THRA, PDPK1, SRC, PIK3R1, ESR1, PIK3CG, SLC9A1, RXRB, RXRA, AKT2, MDM2, MAPK1, PRKACA, TP53, MAPK3
hsa04917	Prolactin signaling pathway	1.04E-11	GSK3B, MAP2K1, SRC, PIK3R1, MAPK14, ESR1, PIK3CG, ESR2, GCK, MAPK10, MAPK8, AKT2, MAPK1, JAK2, MAPK3
hsa04914	Progesterone-mediated oocyte maturation	1.41E-11	MAP2K1, HSP90AA1, PIK3R1, IGF1, MAPK14, PIK3CG, IGF1R, MAPK10, CCNA2, MAPK8, AKT2, CDK2, MAPK1, PGR, PRKACA, MAPK3
hsa05212	Pancreatic cancer	4.93E-11	TGFB2, MAP2K1, PIK3R1, EGFR, TGFBR1, PIK3CG, MAPK10, MAPK8, RAD51, AKT2, MAPK1, TP53, BCL2L1, MAPK3
hsa04068	FoxO signaling pathway	9.15E-11	TGFB2, MAP2K1, PDPK1, INSR, PIK3R1, IGF1, MAPK14, EGFR, TGFBR1, PIK3CG, IGF1R, MAPK10, MAPK8, AKT2, CDK2, MDM2, MAPK1, MAPK3

The article "Network Toxicology Guided Mechanism Study on the Association between Thyroid Function and Exposures to Polychlorinated Biphenyls Mixture" was published in 2022. Journal: Biomed Res Int.

## Data Availability

The datasets used and/or analyzed during the current study are available from the corresponding author on reasonable request.
